The article "Research on Chorus Emotion Recognition and Intelligent Medical Application Based on Health Big Data" was published in 2022. Journal: J Healthc Eng.

# Research on Chorus Emotion Recognition and Intelligent Medical Application Based on Health Big Data

**DOI:** 10.1155/2022/1363690

**Published:** 2022-03-09

**Authors:** Yu Li, Yao Chen

**Affiliations:** School of Music, Sichuan Normal University, Chengdu 610000, China

## Abstract

In chorus activities, the conductor leads chorus members to recreate music works. If you want to interpret music works perfectly with sound, emotion and emotional expression are particularly important. In this paper, a cloud HBD (health big data) integration system based on ensemble learning is designed to realize the high-efficiency and high-precision integration of HBD. An emotional speech database containing three emotions such as pleasure, calmness, and boredom is established, and the corpus problems such as emotional feature analysis and extraction needed for chorus emotion recognition research are solved. It also studies the classification and decision-making in emotional changes, and a DBN (deep belief network) chorus emotion recognition algorithm based on multiple emotional features is proposed. Feature DBN (Deep Belief Network) Chorus Emotion Recognition Algorithm This paper extracts various robust low-level features according to different features' ability to describe emotions and then feeds them into the DBN network to extract high-level feature descriptors. Then, the classification results of ELM (extreme learning machine) are voted and fused with the idea of ensemble learning, and the effectiveness of the algorithm is proved on three public datasets.

## 1. Introduction

Chorus is a collective artistic activity, which emphasizes the commonality and unity of performers. When it comes to unity in chorus, it means not only breathing, articulation, articulation, speed, timbre, volume, and movement but also the unity of emotion and emotional expression [1]. Because in rehearsal and performance, in order to make the expressive force of chorus more perfect, we should not only train basic skills but also be good at mobilizing and unifying the emotions and feelings of chorus members, thus forming the resultant force of collective singing. However, while emphasizing the common features, we often ignore an important issue in music art: emotional expression [2]. This makes the supposed beautiful voice and ideological connotation lack verve and artistic appeal.

Information technology and Internet technology have been widely used in the field of intelligent medical care, and big data provides an opportunity to deeply explore the value of data in the field of intelligent medical care and health. Literature [3] looks at the scenarios and advantages of the application of IoT (Internet of Things), cloud computing, and big data in smart medical health. Literature [4] expounds on the technical route of big data in the field of intelligent medical health from the perspective of methodology. Literature [5] puts forward the life cycle model of smart medical big data and discusses the goals and measures of smart medical big data governance. Literature [6] puts forward a universal intelligent medical information management and service system, and points out the key problems and future research directions of universal intelligent medical computing. Literature [7, 8] put forward a classification method with pitch frequency related information as its main feature, analyze and study four emotional states: fear, anger, sadness, and pleasure, and point out in its research report that the maximum, minimum, and median pitch frequencies are prominent features in speech emotion recognition. Literature [9] in its experimental research, the cepstrum coefficient feature is used as the emotional feature to classify three kinds of emotions, namely sadness, anger, and calmness, and the recognition rate is about 64%, while the accuracy rate of voice samples used by the subjective judgment of people is only 70%. On the basis of statistical analysis of acoustic features related to duration, energy, fundamental frequency, and formant construction of continuous pronunciation, it is proposed that the difference in feature vector between emotional speech and calm speech is taken as an emotional feature vector. Literature [10–12] use principal component analysis to classify pleasure, surprise, anger, and sadness, and the recognition rate is close to 80%. By analyzing the big data of health intelligent medical care, we can find out the correlation and trend among the data, which is helpful to improve the health service and disease exploration process, to conduct disease diagnosis and treatment more scientifically, to improve the efficiency and quality of health intelligent medical care services, and to continuously meet diversified health needs [13]. However, the application of big data in the field of intelligent medical health is still in its infancy, and there is still a lack of general big data framework and standards, which leads to the inability of large-scale application across industries and regions, and the inability to really play the role of big data.

Emotion is an important instinct of human beings. Like rational thinking and logical reasoning ability, it plays an important role in people's daily life, work, communication, transaction processing, and decision making. Based on HBD (health big data), this paper is applied to the emotion recognition of choir for the first time and identifies six basic human emotions, such as joy, anger, surprise, sadness, fear, and calm. The chorus emotion recognition algorithm based on multifeature DBN has the advantages of fast convergence speed, high robustness, and strong global searching ability so as to optimize the connection weights of the neural network. It can not only give full play to the generalization ability of the neural network but also improve the convergence speed and learning ability of the neural network.

## 2. Research Method

### 2.1. HBD Integration System

#### 2.1.1. System Architecture

In some chorus competitions and performances, we hear neat, unified, and beautiful voices without sincere feelings, and the facial expressions of the chorus members are not rich enough, which makes people feel the fly in the ointment. If you want to truly achieve harmony of voice and emotion, you must do a good job of second creation; then, the singer's ideological height, life experience, and artistic accomplishment play a leading role. An excellent chorus player should have rich cultural connotations and literary and artistic accomplishments besides music knowledge and high singing skills. To build a cloud-based HBD integration system, the framework diagram is shown in Figure 1.

The management layer, big data analysis layer, whole cloud HBD integration layer, and whole cloud HBD resource layer constitute a whole cloud HBD integration system. The four layers cooperate with each other to realize the collection, analysis, storage, and operation of the whole cloud HBD.

The interface for users to regulate and use the integrated system is the management operation layer, and the management, regulation, protection, and use of the whole cloud HBD integrated system are realized through the operation of the administrator on this layer [14].

The integrated HBD is stored in the temporary database and metadata of the cloud-wide HBD resource layer and then stored in the cloud-wide HBD integration layer, which is applied to practical application software to complete the integration of cloud-wide HBD based on integrated learning so as to ensure that the cloud-wide HBD resources have higher value embodiment and manageability when integrated [15, 16].

#### 2.1.2. HBD Prediction Method

As chorus art is a form of collective singing, most chorus training emphasizes the common factors of chorus, such as the unity of strength, sound, and expression, to form the resultant force of collective singing. However, while emphasizing generality, emotional expression in music art is often neglected. This makes the sound that should be beautiful and full of ideological connotation lack charm and artistic appeal.

Health informatization has become the core power of innovation and development in the field of big health. Various information systems provide convenient services for the daily work of health and smart medical institutions and at the same time effectively improve their data collection and storage capabilities. Many dynamic nonlinear features are hidden in one-dimensional health sign data, which makes them nonstationary, complex, and unpredictable time series data.

Time series data refers to a series of data values indexed by time. It is common to sample at continuous and equally spaced moments to form a time series. The biggest feature of time series is uncertainty. However, there is a certain mapping relationship within the data. Using intelligent analysis and prediction methods to solve this specific relationship and dig out the potential laws can effectively grasp the future trend of the system.

From a qualitative point of view, if the system parameters and external conditions do not change, then the sampled sequence is stable. However, this kind of analysis is not reliable, and it needs certain statistical characteristics for auxiliary inspection.

For any *m* time series data {*Y*_*t*_}, if its subset {*Y*_*t*_1__,…, *Y*_*t*_*n*__} and subset {*Y*_*t*_1+*m*__,…, *Y*_*t*_*n*+*m*__} are the same, then {*Y*_*t*_} is strictly stationary. The data with strict stationarity have no changing trend. In fact, this kind of data does not exist. Generally, the so-called stationary time series data are weak stationary time series data.

The expectation, variance, and covariance of weakly stationary time series data {*Y*_*t*_} do not change with time [17]. That is,

(1) $$\begin{array}{c} E\left(y_{t}\right)=\mu ,\\ Var\left(y_{t}\right)=\sigma^{2},\\ Cov\left(y_{t},y_{s}\right)=f\left(t-s\right). \end{array}$$

After the time series has passed the stationarity check, the prediction model can be constructed through the relevant fitting model. For nonstationary time series data, it is necessary to process the stationarity and then rebuild the model.

The SARSA (state action reward state action) learning method is a complete state-action transition. When updating the current state action [18], this method does not use the state value function at the next moment but randomly selects actions to update the current state-action space according to a certain probability value and determines the execution action at the next moment when updating, which is the core of the SARSA method [19].The mathematical expression is described as follows:

(2) $$\begin{array}{c} Q\left(s,a\right)\leftarrow Q\left(s,a\right)+\alpha \left[r+\gamma Q\left(s^{\prime },a^{\prime }\right)-Q\left(s+a\right)\right]. \end{array}$$

In the above formula, (*s*, *a*) represents the state action at the current moment, (*s*′, *a*′) represents the state action at the next moment, *r* is the reward obtained after executing the action *a*, and *α* is the step size.

In this paper, a deep reinforcement learning method of SARSA based on “in-strategy” is proposed. The method proposed in this chapter is used to calculate the optimal decision. Let the current state be *s*, *ε* − *greedy* as the selection strategy, the action be *a*, the current action report be *r*, and the next state be *s*′. Then, the current action value function *Q*(*s*, *a*) is described as

(3) $$\begin{array}{c} Q^{*}\left(s,a\right)=E\left[r+\gamma Q\left(s^{\prime },a^{\prime }\right)|s,a\right], \end{array}$$

in which *Q*^*∗*^(*s*, *a*) represents the optimal value of the current value function, and *a*′ represents the optimal action selection at the next moment. Combined with CNN (convolutional neural network), if the network parameter is *λ*, the loss function in the *j* th iteration is defined as

(4) $$\begin{array}{c} L_{j}\left(\lambda_{j}\right)={\left(y_{j}-Q\left(s,a;\lambda_{j}\right)\right)}^{2}, \end{array}$$

in which *y*_*j*_=*r*+*γQ*(*s*′, *a*′; *λ*_*j*−1_). By the differential solution of formula (4), the gradient of loss function can be obtained as follows:

(5) $$\begin{array}{c} \nabla L_{j}\left(\lambda_{j}\right)=\left(r+\gamma Q\left(s^{\prime },a^{\prime };\lambda_{j-1}\right)-Q\left(s,a;\lambda_{j}\right)\right)\nabla Q\left(s,a;\lambda_{j}\right). \end{array}$$

The deep reinforcement learning process and its data flow based on the improved SARSA can be obtained from the formula above.

#### 2.1.3. HBD Interpretation

In order to improve the accuracy and stability of the one-dimensional health sign data prediction model based on deep reinforcement learning, the data interpretation process shown in Figure 2 is designed.

Chorus health data analysis and processing system based on big data can provide health management services for chorus members. Through physical measurement, we can learn about chorus members' physical health status, build an interactive basic service and medical ecological platform [20, 21], and realize interactive sharing of key information between the system and the platform so as to provide efficient personalized physical health services for chorus members and promote optimal management of chorus members' self-health [22].

Because of the multifarious types of indicators, the interface display analysis is based on the body mass index. The function module of weight increase is to increase the physical indicators of chorus members, set the corresponding threshold range reasonably, and dabble in data evaluation standards. In the system, the chorus's physical measurement data, that is, the score calculation, are mainly based on individual indicators and weights, or grades' scoring items and scoring weights, so as to obtain the chorus's total score.

### 2.2. Emotion Recognition of Chorus Staff

Emotion accompanies every moment of human life. About 38% of the information transmitted during human communication is carried by emotions. When people have a natural oral conversation, they not only convey the voice but also convey the speaker's emotional state, attitude, and intention.

The application of “emotion” in chorus can not only resonate with chorus members and audience but also realize the artistry of the chorus. In essence, emotional unity is a part of chorus unity. In the process of chorus rehearsal, we must follow the principle of chorus unity. The realization of chorus unity plays a very important role in the whole chorus rehearsal process.

In the process of chorus rehearsal, the chorus members should deeply understand the connotation of music and fully reflect the different attributes of each song so as to realize the resonance between the chorus members and the audience. Only in this way can we give full play to the artistry of chorus and achieve a perfect artistic realm.

This study mainly studies the algorithm of chorus emotion recognition. With the help of the excellent performance of neural network technology and the complementarity between different voice features, the idea of ensemble learning is introduced to complete the task of voice signal recognition under different emotions.

#### 2.2.1. Emotional Feature Analysis

In chorus rehearsal, the commander should command the chorus's singing work on the one hand and interpret the music works on the other hand. Before chorus rehearsal, the commander should fully do desk work, get a deep understanding of the works of singing tracks and the background of the times, content forms, and cultures in which the singing tracks are produced, and put himself in another's shoes, understand the aesthetic requirements of songwriters for music, and realize the recreation of music on this basis.

Speech energy is one of the most important features in prosody, which is mainly determined by the vibration amplitude of the signal and reflects the strength of sound. In real life, people can feel that when a person expresses sad feelings, his voice is generally vague and low, while when he expresses happy and angry feelings, his voice is generally loud and bright. Therefore, different emotional voices have obvious differences in speech energy characteristics.

In view of which features in speech signals can effectively reflect emotion, researchers have carried out a lot of research from the perspectives of psychology and phonetic linguistics, but at present, they pay most attention to two types: prosodic features and sound quality features. This kind of feature and its derived parameters are most widely studied and applied in chorus emotion recognition. Sound quality features mainly refer to the timbre and spectrum of speech, so they are also called segmental features, which reflect the change of glottal wave shape during pronunciation (Figure 3).

If music only has notes and rhythms, it is just a shell. Only by giving rich emotions, the expression of music can be fuller and more perfect. Emotion and emotional expression run through the chorus. As chorus conductors, we should fully realize the importance of emotions and emotional expressions when interpreting chorus works and be good at unifying the emotions of members in the chorus process so as to make the chorus art more perfect.

Prosodic features and phonetic features are not isolated. Literature [23, 24] show that there is a certain correlation between prosodic features of speech signals and three emotional dimensions (valence dimension, activation dimension, and control dimension). Among them, the activation dimension is obviously related to prosodic features, and emotional states with similar activation dimensions have similar prosodic features, which are easy to be confused. By judging voiced and unvoiced speech signals, unnecessary calculation of the autocorrelation function of unvoiced frames can be effectively eliminated, and the calculation amount of pitch detection can be reduced.

The purpose of pitch detection preprocessing is to improve the accuracy of pitch detection by the autocorrelation method, which mainly includes band-pass filtering and nonlinear transformation. This paper only introduces the nonlinear transformation method. Commonly used nonlinear transformation methods include center clipping and three-level clipping. In this paper, the towel-center wave elimination method is adopted, and formula (6) is used as the central clipping function expression:

(6) $$\begin{array}{c} y\left(n\right)=\left\{\begin{array}{cc} x\left(n\right)-L, & x\left(n\right)>L,\\ 0, & \left|x\left(n\right)\right|\leq L,\\ x\left(n\right)+L, & x\left(n\right)<-L, \end{array}\right. \end{array}$$

where *y*(*n*) is the output of the central clipping function, and *x*(*n*) is the input, which is the amplitude of *n* sample points in a frame of speech signal, and is the clipping level, which is a constant related to the maximum amplitude of the current frame. Usually, 60%–70% of the maximum amplitude is taken, and this paper takes 0.68.

The function definition of three-level clipping is

(7) $$\begin{array}{c} y\left(n\right)=\left\{\begin{array}{cc} 1, & x\left(n\right)>L,\\ 0, & \left|x\left(n\right)\right|\leq L,\\ -1, & x\left(n\right)<-L. \end{array}\right. \end{array}$$

Comparing the expressions (6) and (7), it can be seen that the three-level clipping is a correction based on the central clipping, and the sample points exceeding the clipping level are assigned as 1 or -1, which can effectively reduce the multiplication in the calculation process of the autocorrelation function.

In order to analyze the relationship between formant-related features and emotional state, we extracted the first formant one by one from the emotional voice database. On this basis, the statistical characteristics of the first formant in different emotional states are statistically analyzed.  Figure 4 shows the statistical analysis results of the mean value, dynamic range, and change rate of the first resonance peak.

It can be seen from the figure that the mean value of the first formant of pleasure and boredom is higher than that of the dynamic range, while the change rate is pleasure < calm < boredom, and the difference between the change rates of boredom and pleasure emotions is obvious.

#### 2.2.2. Emotion Recognition of Chorus Based on Multifeature DBN

People can fully express their true feelings and thoughts through music. Emotion can be said to be the basic attribute of music. If a song lacks emotional integration, even if it has the best singing skills, it will be difficult for the audience to resonate with it. As music performers, musicians should fully tap the emotions in music, accurately understand the author's thoughts and feelings, and on this basis, organically integrate their feelings with music and recreate chorus music. Only in this way we can fully express the image that music wants to create and arouse the audience's resonance.

In this paper, we consider adopting the method of deep learning, extracting higher-level descriptors to represent more abstract concepts, and extracting more robust feature parameter factors through the multilevel representation of speech signals. The deep learning method has created the latest records in image processing, target location, detection, and other recognition and classification tasks, and DBN is one of the most representative networks.

The Boltzmann machine is an early component of the neural network, and its neurons are divided into two parts: explicit layer and implicit layer. The explicit layer is the input and output layer, which indicates the transmission of data, while the hidden layer is equivalent to the need to adjust the data in the transmission process, adding weight. The standard Boltzmann machine is a fully connected graph, and the complexity of the training network is very high. Therefore, in practice, the RBM (restricted Boltzmann machine) shown in Figure 5 is usually used for simplification.

The construal divergence (CD) algorithm is often used to train constrained Boltzmann machines. Assuming that there are *d* neurons in the explicit layer and *q* neurons in the hidden layer in the network, let *v* and *h* represent the state vectors of the explicit layer and the hidden layer, respectively; then, because there is no connection in the same layer, there are

(8) $$\begin{array}{c} P\left(v|h\right)=\overset{d}{\underset{i=1}{\prod }}P\left(v_{i}|h\right),\\ P\left(h|v\right)=\overset{q}{\underset{j=1}{\prod }}P\left(h_{j}|v\right). \end{array}$$

The connection weight update formula is

(9) $$\begin{array}{c} \Delta w=\eta \left(vh^{T}-v^{\prime }h^{\prime T}\right). \end{array}$$

DBN (deep belief network) is connected by multiple RBM stacks, which can be trained effectively in a hierarchical way. Therefore, DBN has a strong learning ability and can learn high-level feature descriptors which are beneficial to the emotional recognition of chorus, as shown in Figure 6.

Firstly, it trains the first RBM with training samples and then uses the output of the first RBM as the input of the second RBM. Similarly, the output of the second RBM is used to train the third RBM. After each layer is pretrained, the whole network is trained by the BP algorithm.

In this way, we can build a deep network model and then use the network model to obtain more robust high-level feature descriptors from low-level features.

In order to extract higher-level feature descriptors in speech emotion and ensure the diversity of base classifiers, inputting multiple features into the DBN network can solve the above problems. Therefore, this paper proposes a multifeature DBN method for chorus emotion recognition, which is composed of multifeature selection, DBN, and ELM (extreme learning machine) within the framework of set learning. The system framework is shown in Figure 7.

In this paper, we need to use spectrum sequence context (SSC) feature, power-normalized cepstral coefficient (PNCC), rhythm (Rhys) feature, Mel cepstrum coefficient (MFCC), and perceptual linear prediction (PLP), and then input these multiple features into the DBN network after feature selection so as to extract higher-level feature descriptors and create a better classifier.

Traditional hand-designed features do not perform well in emotion recognition tasks, mainly because they are low-level features, and it is difficult to fully describe the deep-seated information hidden in emotions [25]. Therefore, with the help of deep learning methods, a variety of traditional features are integrated with the DBN network to achieve better recognition results in emotion recognition tasks.

## 3. Discussion and Analysis

### 3.1. Comparison of Prediction Results

Based on the historical blood pressure data in the database of Literature [22], 221 experimental individuals, aged between 60 and 75 years, were preliminarily screened out. Predicting the blood pressure trend of these kind of people can help them control their blood pressure, guide their medication, and provide early risk warnings for some diseases.

Figure 8 shows the comparison between the actual value of blood pressure time series data and the prediction result of the model, and Figure 9 shows the error prediction model.

It can be seen from Figures 8 and 9 that the ARIMA-SVM model has higher prediction accuracy than the traditional ARIMA model and overcomes the limitations of the single model. Q-learning-based deep reinforcement learning and SARSA-based deep reinforcement learning are superior to the former two in high-dimensional spatial prediction, so the prediction accuracy is higher than the former two. Especially, the deep reinforcement learning method based on SARSA learning can fully express the hidden information in the original time series data of blood pressure.

### 3.2. Efficiency of HBD Integration

When the storage capacity of experimental big data is increasing, the two systems integrate the HBD efficiency of experimental logistics companies. The results are shown in Figure 10.

As can be seen from Figure 10, this system is highly efficient in integrating the whole cloud HBD.

The results of testing the concurrency of HBD integrated in this paper are shown in Figure 11.

According to the analysis of Figure 11, with the increase of time, the system in this paper is much larger than the HBD integration system based on IoT in processing the whole cloud HBD, which shows that the system in this paper has higher performance in processing the whole cloud HBD.

### 3.3. Analysis of Chorus Emotion Recognition

In order to verify the effectiveness of the spectral context features proposed in this paper in chorus emotion recognition, we compare the classical MFCC features and the combination of MFCC and delta features with the spectral context features on Berlin Emo-DB, SAVEE, and CASIA datasets, respectively. ELM classification is adopted in the classifier, with the number of hidden nodes being 6,000 and the activation function being hardlim.  Figure 12 shows the comparison of the emotion recognition accuracy of different classifiers (speaker dependent).

In Figure 12, we compare the algorithm in this paper with KNN, SVM, ELM, single-layer DBN network (SLDBN), and double-layer DBN network (DLDBN). The experimental results show that the accuracy of the algorithm in this paper is greatly improved than the above methods, which shows that the algorithm in this paper can more effectively classify and recognize speech emotions.

In this experiment, 8 chorus samples were randomly selected from the Berlin Emo-DB dataset as the training set and the remaining 2 chorus samples as the test set. In order to avoid the error caused by the randomness of samples, we chose to repeat the experiment 5 times and calculate the average recognition accuracy.  Figure 13 shows the comparison of emotion recognition accuracy of different classifiers (speaker independent).

Through Figure 13, we find that in the speaker independent experiment, the algorithm in this paper is compared with KNN, SVM, ELM, single-layer DBN network (SLDBN), and double-layer DBN network (DLDBN). The experimental results show that the algorithm in this paper is better than the above methods. Both have improved, indicating the effectiveness of the algorithm in this paper for the emotion recognition of chorus personnel.

## 4. Conclusion

If music only has notes and rhythm, it is just an empty shell. Only by giving rich emotions can the expression of music be fuller and more perfect. Emotion and emotional expression run through the chorus. The research work of emotional feature analysis and extraction is carried out in the established emotional voice database, and the changing rules of energy, fundamental frequency, formant, and other features in different emotional states are observed and analyzed. According to the statistical analysis results, the global statistical emotional features with emotional discrimination are selected and extracted. In this paper, according to the different abilities of different features to describe emotions, various robust low-level features are extracted, and then they are fed into the DBN network to extract high-level feature descriptors. Then, the ELM classification results are voted and fused with the idea of ensemble learning, and the effectiveness of the algorithm is proved on three public datasets.

## Figures and Tables

**Figure 1:** Framework diagram of HBD integration system.

**Figure 2:** Data interpretation process.

**Figure 3:** Harmonic noise ratio characteristics of emotion.

**Figure 4:** Comparison of the first formant characteristics of three emotions.

**Figure 5:** Restricted Boltzmann machine.

**Figure 6:** DBN structure diagram.

**Figure 7:** Flowchart of chorus emotion recognition based on multifeature learning.

**Figure 8:** Comparison between actual values and model prediction results.

**Figure 9:** Comparison of final prediction errors of four models.

**Figure 10:** Efficiency of HBD integration.

**Figure 11:** Test effect of integration system concurrency.

**Figure 12:** Comparison of emotional recognition accuracy of different classifiers.

**Figure 13:** Comparison of emotional recognition accuracy of different classifiers.

## Data Availability

The data used to support the findings of this study are included in this paper.

## References

[1] Zhan K. (2020). Sports and HBD system based on 5G network and Internet of Things system. *Microprocessors and Microsystems*.

[2] Choi S.-Y., Chung K. (2020). Knowledge process of health big data using MapReduce-based associative mining. *Personal and Ubiquitous Computing*.

[3] Yang T., Yuan G., Yan J. (2021). Health analysis of footballer using big data and deep learning. *Scientific Programming*.

[4] Xing W., Bei Y. (2019). Medical HBD classification based on KNN classification algorithm. *IEEE Access*.

[5] Barik R. K., Dubey H., Mankodiya K. (2019). GeoFog4Health: a fog-based SDI framework for geospatial HBD analysis. *Journal of Ambient Intelligence and Humanized Computing*.

[6] Zhou S., He J., Yang H., Chen D., Zhang R. (2020). Big data-driven abnormal behavior detection in healthcare based on association rules. *IEEE Access*.

[7] Christie M., Lisa J. (2019). The intersection of mobile health and nursing knowledge: big data science. *Computers, informatics, nursing: CIN Plus*.

[8] Han K., Zhang L., Tian Z., Gu Y. (2021). Human muscle measurement and big data health based on wireless sensors. *Microprocessors and Microsystems*.

[9] Raja R., Mukherjee I., Sarkar B. K. (2020). A systematic review of healthcare big data. *Scientific Programming*.

[10] Yu H. Q., Dong F. (2019). Semantic lifting and reasoning on the personalised activity big data repository for healthcare research. *International Journal of Web Engineering and Technology*.

[11] Khan B., Naseem R., Shah M. A. (2021). Software defect prediction for healthcare big data: an empirical evaluation of machine learning techniques. *Journal of Healthcare Engineering*.

[12] Xie B., Kim J. C., Park C. H. (2020). Musical emotion recognition with spectral feature extraction based on a sinusoidal model with model-based and deep-learning approaches. *Applied Sciences*.

[13] Schmidt T., Schlindwein M., Lichtner K., Wolff C. (2020). Investigating the relationship between emotion recognition software and usability metrics. *I-Com*.

[14] Jiaqi W., Liu H., Wang B. (2019). Extreme learning machine for emotion recognition of tactile gestures. *Caai Transactions on Intelligent Systems*.

[15] Slimani K., Kas M., Merabet Y. E., Ruichek Y. (2020). Local feature extraction based facial emotion recognition: a survey[J]. *International Journal of Electrical and Computer Engineering*.

[16] Nashipudimath M. M., Pillai P., Subramanian A., Nair V. (2021). Voice feature extraction for gender and emotion recognition. *ITM Web of Conferences*.

[17] Deepika C. (2020). Speech emotion recognition feature extraction and classification. *International Journal of Advanced Trends in Computer Science and Engineering*.

[18] Lawrence S., Anjum T., Shabani A. (2021). Improved deep convolutional neural network with age augmentation for facial emotion recognition in social companion robotics. *Journal of Computational Vision and Imaging Systems*.

[19] Hamsa S., Iraqi Y., Shahin I., Werghi N. (2021). An enhanced emotion recognition algorithm using pitch correlogram, deep sparse matrix representation and random forest classifier. *IEEE Access*.

[20] Luo H., Han J. (2020). Nonnegative matrix factorization based transfer subspace learning for cross-corpus speech emotion recognition. *IEEE/ACM Transactions on Audio, Speech, and Language Processing*.

[21] Lin W. C., Busso C. (2021). Chunk-level speech emotion recognition: a general framework of sequence-to-one dynamic temporal modeling. *IEEE Transactions on Affective Computing*.

[22] Mansouri-Benssassi E., Ye J. (2020). Synch-graph: multisensory emotion recognition through neural synchrony via graph convolutional networks. *Proceedings of the AAAI Conference on Artificial Intelligence*.

[23] Zang H., Foo S. Y., Bernadin S., Baese A. M. (2021). Facial emotion recognition using asymmetric pyramidal networks with gradient centralization. *IEEE Access*.

[24] Nair V., Pillai P., Subramanian A., Nair V. (2021). Voice feature extraction for gender and emotion recognition. *International Journal on Recent and Innovation Trends in Computing and Communication*.

[25] Yan G., Sha R. (2020). Autonomous learning of foreign language based on facial emotion recognition and cloud computing. *Journal of Intelligent and Fuzzy Systems*.

